# Single image super-resolution via Image Quality Assessment-Guided Deep Learning Network

**DOI:** 10.1371/journal.pone.0241313

**Published:** 2020-10-29

**Authors:** Zhengqiang Xiong, Manhui Lin, Zhen Lin, Tao Sun, Guangyi Yang, Zhengxing Wang

**Affiliations:** 1 Electronic Information School, Wuhan University, Wuhan, China; 2 State Key Laboratory of Information Engineering in Surveying, Mapping, and Remote Sensing, Wuhan University, Wuhan, China; 3 Computer and Science School, Wuhan University, Wuhan, China; 4 State Key Laboratory of Bridge Structure Health and Safety, Wuhan, China; University College London, UNITED KINGDOM

## Abstract

In recent years, deep learning (DL) networks have been widely used in super-resolution (SR) and exhibit improved performance. In this paper, an image quality assessment (IQA)-guided single image super-resolution (SISR) method is proposed in DL architecture, in order to achieve a nice tradeoff between perceptual quality and distortion measure of the SR result. Unlike existing DL-based SR algorithms, an IQA net is introduced to extract perception features from SR results, calculate corresponding loss fused with original absolute pixel loss, and guide the adjustment of SR net parameters. To solve the problem of heterogeneous datasets used by IQA and SR networks, an interactive training model is established via cascaded network. We also propose a pairwise ranking hinge loss method to overcome the shortcomings of insufficient samples during training process. The performance comparison between our proposed method with recent SISR methods shows that the former achieves a better tradeoff between perceptual quality and distortion measure than the latter. Extensive benchmark experiments and analyses also prove that our method provides a promising and opening architecture for SISR, which is not confined to a specific network model.

## 1. Introduction

Despite the rapid development of imaging technology, imaging devices still have limited achievable resolution due to several theoretical and practical restrictions. Super-resolution (SR) technology provides a far promising computational imaging approach to generate high-resolution (HR) images via an existing low-resolution (LR) image or image sequences, which have been widely applied in video surveillance, medical diagnostic imaging, as well as radar imaging systems. SR has two main categories, namely, single image SR (SISR) and multi-frame image SR (MISR) [1]. SISR is practical in many aspects because it has unlimited amount of LR input images [2]. For this reason, this study mainly focuses on the SISR problem.

SISR is an underdetermined inverse problem, and, thus, is relatively challenging because a given LR input image may have multiple solutions based on various texture details in its corresponding HR image. Two problems need to be addressed to generate high-quality SR images. The first problem refers the unsatisfactory edge preservation and texture restoration caused by insufficient regularized constraints given that a single image provides very limited feature information. The second problem refers the difficulty in the quantitative evaluation of the estimated parameters because of the inability to measure their ground truth [3–5].

In recent years, deep neural networks (DNN) have been widely used in SR and have demonstrated superior performance [6, 7]. Several quintessential methods, such as non-uniform interpolation, frequency domain, and machine learning-based reconstruction approaches, have been developed for SR. Although these methods can provide optimal or near-optimal images that increase the resolution, they cannot guarantee detail enhancement, such as loss of high-frequency information and edge blur.

To solve these problems, deep learning-based SR methods are developed given that the mapping relations of image feature from LR to HR can be fully explored, and the reconstruction results have remarkable robustness and stability in multiple scale spaces [8,9].

According to the form of the loss function, existing deep learning-based SR methods fall largely into two categories: 1) *Absolute loss (AL)-based methods* [10–13]. AL-based methods mainly focus on improving the quantitative indicator of IQA and generally take the forms of MSE or MAE. 2) *Perceptual loss (PL)-based methods* [14–17]. PL-based methods are imported to avoid excessive smoothing, and perceived quality has been the primary concern in the subsequent approaches.

Blau [18] proved that the distortion and perceptual quality of an image were at odds with each other. Thus, algorithms with less distortion generally suffer from poor perceived quality, and vice versa. To satisfy diverse demands, we cannot simply conclude that one is more important than the other. In practical applications, the excellent performance of one indicator (absolute or perceived quality) or determining a compromise approach is likely to be given attention.

Recently, PL has elicited increasing attention given that images have been observed by humans eventually. Nevertheless, perception features are extracted by preliminary trained net among the existing methods, thereby causing the inefficiency of the extracted features. This phenomenon is mainly caused by the different datasets that are used by the training and SR nets. Therefore, a SISR model, which integrates image quality assessment (IQA) to SR is proposed. Specifically, perception features are extracted from SR results by IQA net to calculate corresponding PL. After that, PL is fused with original pixel loss, thereby leading to the remarkable convergence of the SR parameters that are balanced between human perception and distortion measure.

In our work, IQA network is injected to guide the training of SR net. On the one hand, the IQA net, which is different from SR generative adversarial network (SRGAN) [19], adaptively adjusts itself to a new distribution of input images that avoid an explicit adversarial training. On the other hand, visual geometry group (VGG) [20] and discriminator networks are designed and incorporated with each other. This strategy has dramatically reduced the computing resource while preventing over-fitting problems. The specific contributions of this study are presented as follows:

- An IQA-guided SISR model is proposed creatively using DL networks. Unlike existing DL-based SR algorithms, an IQA net is used to guide the adjustment of SR net parameters and prevent the over-fitting problems.
- We establish an interactive training mechanism via cascaded network, where the IQA net acts as a supervisor when constructing loss function of the SR net, and thus solve the problem of heterogeneous datasets used by IQA and SR networks.
- The approach in this paper is proved to achieve a nice tradeoff between perceptual quality and distortion measure by extensive qualitative and quantitative experiments, taking into account of both absolute pixel loss and visual effects.
- We propose a promising and opening architecture, which is not confined to a specific net model.

The baseline of SR net is expected to be adjusted flexibly according to practical requirements (e.g. Using a generator with better net architecture to obtain improvements in network performance, or selecting another lightweight net architecture to promote the efficiency of the network).

The remainder of this work is organized as follows. Section 2 presents the related works. Section 3 elaborates the net structure of the proposed method. Section 4 presents the experimental results. Section 5 draws the conclusion.

## 2. Related works

### 2.1. Super-resolution

Deep learning technique has gradually become the mainstream in SR field with the rapid development of parallel computing. Conventional methods, including interpolation, frequency domain, and machine learning-based reconstruction approaches, have achieved high reconstruction efficiency [9,21]. However, these methods exhibit limitations in predicting detailed, realistic textures. SR results from deep learning methods outperform those from other approaches in PSNR and perceptual evaluation given the inherent ability of SR to extract high-level features [4,22].

Section 1 highlights the two main SR approaches derived from deep learning, namely, AL-based and PL-based methods. To facilitate understanding, we review several major works of these methods briefly.

#### AL-based SR methods

Although deep networks improve the accuracy of the SR results [10–13], problems, such as over-fitting and large model, appear. Subsequently, deep recursive convolutional network (DRCN) [14], where network depth is increased without introducing new parameters for additional convolutions by using a very deep recursive layer with up to 16 recursions, is proposed to solve these problems. Lim [15] developed an enhanced deep SR network (EDSR) for SISR and achieved a performance that exceeded those of the state-of-the-art SR methods via optimization by removing unnecessary modules in the conventional residual networks (ResNet) [16]. Inspired by ResNet, VDSR, and DRCN, a deep recursive residual network (DRRN) with relatively deep network structure is designed by adjusting the architecture of existing ResNet. In this network, residual learning is adopted globally and locally to mitigate the difficulty of training, and recursive learning is used to control the model parameters. Extensive benchmark assessment shows that DRRN significantly outperforms state-of-the-art methods in SISR. Zhang *et al*. [17] presented a very deep residual channel attention network (RCAN), where a residual in residual structure is proposed to form a very deep network. The main network focuses on learning high-frequency information by short skip connections, thereby promoting the system performance.

The key idea of these methods is to minimize the MSE between SR and HR images. However, MSE essentially focuses on pixel loss. Consequently, dealing with uncertainty in restoring high-frequency details is difficult. Specifically, images generated from MSE face the over-smooth problems, and thus, cannot match up to the human visual system [23]. Considering the subjective image quality, perception-based constraints are introduced to act as the loss functions.

#### PL-based SR methods

The SRGAN proposed by [19] was considered the opening research of the PL-based SR approach. Perceptual loss was presented for the first time in the field of SISR. Instead of the typically used per-pixel loss, a feature reconstruction loss was introduced to allow the transfer of semantic knowledge from the pre-trained loss network to the SR network. The results show that this work is effective in reconstructing fine details, thereby leading to positive visual results. In [24], the authors enhanced the vein features by adding generative adversarial network (GAN) loss. The idea is to constrain the SR images to satisfy the regulation of natural images. Sajjadi [23] introduced texture matching loss, which generated abundant texture information, on the basis of [25]. Wang [26] proposed a stereo SR network to integrate the information from a stereo image pair for SR, which effectively captures stereo correspondence to improve SR performance. Guo [27] designed an ORDSR network by using DCT, thereby achieving state-of-the-art SR image quality with less parameters than most deep CNN methods. Cao [28] developed a multi-scale residual channel attention network, considering that the increase in network depth resulted in the difficulty of training the network. The network exploited the image feature with conventional kernels of different sizes and used a channel attention mechanism to recalibrate the channel significance of feature mappings adaptively. The experiments on the benchmark dataset show that the proposed method can compete with the state-of-the-art SR methods.

Since images are observed by humans eventually, PL has been paid much attention recently. Nevertheless, perception features are extracted by preliminary trained net and different datasets are used between training and testing nets among most existed methods, leading to the ineffectiveness of the extracted features. Besides, few of the methods mentioned above take into account of both perceptual quality and distortion measure of the SR result simultaneously. To address this issue, IQA is introduced to our work. The detailed network architecture will be explained in Section 3.

### 2.2 Image quality assessment

IQA has become the basic research of the related areas of image processing, the assessment results of which act as the reference indicator of the image processing system [29]. IQA, as a crucial step in image processing, can clearly reflect image distortion, serve as the basis for image automatic filtration, and be considered as the network feedback to guide parameter adjustment. In general, IQA methods fall into two categories, namely, full-reference (FR) and no-reference (NR) methods, depending on whether a reference image is required [30].

FR-IQA methods refer to the quality assessment of distorted images by comparing with the original image, which is an undistorted version of the same image. The simplest approach to measure image quality is by calculating the PSNR and the structural similarity index metric (SSIM) [31]. However, PSNR and SSIM do not always correlate with human visual perception and image quality. Other IQA methods were proposed to address the limitation of PSNR and SSIM. IQA metrics, including visual information fidelity (VIF) [32], Fast SSIM [33], information fidelity criteria (IFC) [34], multi-scale structural similarity (MS-SSIM) [35], and mean deviation similarity index (MDSI) [36], correlate well with human perception.

NR-IQA has experienced two phases in its development course, namely, machine learning and deep learning. In general, learning-based methods establish the mapping relations between image features and quality. Moorthy [37] first applied machine learning to IQA, in his work, support vector machine (SVM) and natural scene statistics (NSS) were incorporated with each other to achieve favorable results, and their combination was called BIQI. Subsequently, many different methods, including DIIVINE [38], BRISQUE [39], BLIINDS-II [40], and IL-NIQE [41] were introduced gradually. Given the difficult extraction of high-dimensional features for machine learning as the dataset’s scale increases rapidly, deep learning technique is used for IQA. NR-IQA via deep learning (DLIQA) is an innovative work in this field [42]. The author suggested the extraction of multilevel representations from a very deep DNN model for learning an effective NR-IQA method. Subsequently, some other typical DNN, including CNNIQA [43], DeepIQA [44], BIECON [45], dipIQA [46], RankIQA [47], and Hallucinated-IQA [48], were adopted to develop NR-IQA methods. These networks are designed to extract features automatically, and the corresponding mathematical methods are derived. In addition, an end-to-end training approach maps the input images to image quality score output.

NR-IQA methods provide quality images without the need for any reference image or features. The quality measure totally depends on the nature of human visual system because of the absence of reference images [49]. For this reason, NR-IQA is applied in our IQA net.

## 3. Proposed methods

In this section, we describe the proposed deep networks, and the model architecture of which is displayed in Fig 1. Our method consists of two components, namely, SR and IQA networks. SR network intends to generate SR images, and IQA network is used to assess the quality of those input images (*e*.*g*., reconstructed SR images). These networks are creatively cascaded with each other in our work, in order to promote the performance and robustness of SISR network. Specifically, SR images produced by the SR network are imported to IQA network, which outputs the image quality scores. Meanwhile, this image quality indicator is regarded as feedback to SR structure, which guided the training of SR network.

**Fig 1:** Framework of the proposed method, in which SR images produced by the SR network are imported to IQA network, and IQA network outputs the image quality scores in return.

### 3.1 Network structure

#### IQA network

IQA, which serves as feedback, should not only be derivable but also possess appropriate number of network layers. With respect to relatively shallow architectures, such as CNNIQA [44], extracting sufficient feature information is difficult. Relatively deep architectures, such as Hallucinated-IQA [48], face the difficulty of training and consume substantial memory. When coupled with other networks, a very deep architecture would be extremely difficult to design and use. As shown in Fig 2, an improved DeepIQA (DeepIQA has two versions: FR version and NR version, we apply NR version in this work) is used as the IQA net in our work. The figure shows that the feature extraction is realized by cascading convolutional layers in five levels, with increasing channel numbers of 32, 64, 128, 256, and 512. Each level contains two convolutional layers with identical output channel number. The batch normalization layer and the activation function are adopted to connect two adjacent convolutional layers. Strided convolutions are used to reduce the image resolution each time, and the number of features is doubled. Two fully connected (FC) layers are used to map the features obtained from the convolutional layers. The leaky ReLU function [50] is added between the FC layers, and the Sigmoid function [51] is used to limit the output within the range of 0 *−* 1.

**Fig 2:** Architecture of the IQA net, where the feature extraction is realized by cascading convolutional layers in five levels.

Compared with the NR version of DeepIQA, the proposed IQA network is advanced in the following seven aspects:

- All the max pooling layers are substituted by strided convolution layers to avoid gradient instabilities, preventing generation of artifact.
- To avoid gradient sparseness [24], Leaky ReLU is used to take the place of ReLU, and *α* is set to 0.2.
- Since IQA network serves as providing feedback to guide parameters adjustment, the structure of IQA network should not be too complex. To save memory, the first and second down samplings are conducted on the factor of *×*4 (the size of the corresponding convolution kernel is 5 × 5), and the others are achieved on the factor of ×2 (the size of the corresponding kernel is 3 × 3).
- Batch normalization is considered, following each convolution layer to accelerate convergence.
- The brightness range of input images is normalized to [0, 1] by $\hat{I}=I/255$, fitting the feature extraction.
- Instead of the patch size of 32 *×* 32, our method receives patches with the size of 256 *×* 256 as the input to eliminate the boundary effects caused by image blocking.
- Sigmoid function is used to limit the output range between 0 and 1, rendering the output value as probability, thereby resulting in the convenient building of loss functions.

The improved network structure is shown in Fig 2. Feature maps at different depths correspond to varied abstraction levels, representing features of the input image in different dimensions. For convenience, we consider *fli* as the feature map out of the last convolution layer prior to the *i*-th downsampling layer.

#### SR network

To ensure the feasibility of the proposed method, the same structure as EDSR [15] is adopted in this work. EDSR has reduced unnecessary blocks in vanilla ResNet [16], enhancing the performance with a compact model structure. Residual scaling is adopted for ease of stable training of larger models. As shown in Fig 3, the network consists of 16 residual blocks and 64 filters, which ensure that multi-level features can be shared to boost the performance.

**Fig 3:** Architecture of the SR net, the network consists of 16 residual blocks and 64 filters, which ensure that multi-level features can be shared to boost the performance.

### 3.2 Interactive training strategy

Two problems should be tackled in designing a cascade SR network using SR and IQA network, as follows: 1) the existing IQA dataset is extremely small to provide sufficient training samples. Thus, the IQA network should be provided with unsupervised training or self-supervised training. Inspired by RankIQA [47], the pairwise ranking hinge loss is introduced to create training labels dynamically, overcoming the shortcomings of insufficient samples; 2) the IQA network acts as a supervisor in cascaded network when constructing loss function of the SR network. Consequently, the output distribution from the SR net must be covered by the input distribution of the IQA net. To achieve this result, we designed an interactive training mechanism considering feature stability and effectiveness of the IQA features, thereby improving the overall performance.

To ensure that the IQA network can deal with all the SR images generated from the SR network, an intuitive idea would be alternate training. Specifically, we initially train the IQA network for *k* iterations and then use the obtained stable features to guide the training of the SR network for one iteration. Then, the new output of the SR network is fed into the IQA network to calculate losses as well as gradients, accounting for another *k* iterations of training of the IQA net. Evidently, this solution is time consuming when *k* is a large number. In addition, the gradient descent direction provided by the SR net tends to be transient because the parameters of the IQA net update almost continuously. To avoid this condition, we propose a new training solution, where the SR network is trained *n* times after the *k*-time iterative training of the IQA network.

The balance between feature stability and feature effectiveness should be considered. On the one hand, more effective features ensure that the parameters of the SR network converge to an optimum; on the other hand, more stable features guarantee the steady convergence of the SR network. Hence, the selection of *k* and *n* is crucial. In this work, they were determined experimentally.

#### Training of SR network

The parameters of the IQA network are fixed during the SR training. The output from the SR network and the original HR image are placed into the IQA network for perceptive feature extraction. We calculate the similarity between SR and HR images on different feature layers to establish the loss function in the perception level (namely, reconstruction of perceptual loss). In addition, the pixel loss (content loss) between SR and HR images is computed to evaluate the image distortion. Then, a joint loss function is obtained by weighted combination of these losses, which are used to optimize the training performance of the SR network.

#### Training of IQA network

Provided that the parameters of SR network are fixed, we estimate a margin with an FR-IQA method, considering the reconstructed SR result and the HR labels as inputs. Then, the pairwise ranking hinge loss is figured out with a specified margin, enabling self-supervised learning of the IQA network.

#### Alternate training

The results from the IQA network are used to guide the training of the SR network. Thus, the features extracted by the IQA network must be reliable to provide accurate reference information for SR network.

The parameters of the IQA network are fixed during the training of the SR network. Thus, reckoning the IQA features as stable is reasonable. Under this condition, the convergence direction of SR should also be steady. However, the distribution of generated SR images fluctuates as the training continues, deviating from the original distribution gradually.

On the contrary, when the parameters of the SR network are fixed, the assessment ability of the IQA net increases. In other words, the features extracted by the IQA net are more adaptable to the distribution of the input images. Thus, the IQA network can possibly fail to adapt to the newly generated input distributions if the parameters of the SR network are updated rapidly, thereby leading to poor effectiveness. On the contrary, frequent update of the parameters of the IQA network results in difficulty of convergence of the SR network.

Each time of alternate training between the SR network and the IQA network is referred to as a training phase in this work. Then, the two networks should be maintained in the transition state between two phases to allow the IQA net to effectively fit to the output distribution of the SR net during the previous phase. Moreover, the output of the SR net should not be excessively far from its most recent distribution.

### 3.3 Loss functions

To improve the performance of the SR network and ensure that the IQA net effectively guides the training of the SR network, an appropriate loss function should be designed. The loss functions of SR and IQA are discussed as follows.

#### Loss function for SR net

In accordance with the requirements of joint training, the loss function for SR network is formulated as follows:

$$\begin{array}{c} L_{SR}=w_{0}MAE(I^{SR},I^{HR})+\sum_{i=1}^{5}w_{i}\|G(\phi_{i}(I^{SR})),\phi_{i}(I^{HR})){\|}_{F} \end{array}$$ (1)

where *I*^*SR*^ is the SR image, *I*^*HR*^ represents the reference HR image, G denotes the perceptual loss function of IQA net, and *wi*(*i* = *0*, *1*, *2*, …, *5*) is the weight coefficient of loss function. The first term of this function is essentially the content reconstruction loss. Content loss ensures the consistency of content by minimizing the MAE between the SR and HR images. The second term stands for the perceptual loss constructed from various feature layers of the IQA network. To better capture the texture details, the strategy in [23] is considered, where we regard the texture feature as style feature of local blocks and utilize a patch-wise style reconstruction loss. Following the configuration in [23], the patches with the size of 16 *×* 16 are used for texture loss calculation. We use the feature maps that resulted from the convolution layers prior to the first three down-sampling layers to compute the texture loss, denoted as *fl1*, *fl2*, and *fl3*, because much more high frequency information lie in shallow and middle level features.

#### Loss function for IQA net

The deficiency of the training samples is one of the major problems faced by deep learning-based IQA. On the one hand, humans more easily distinguish image quality via comparison of a given image pair than evaluate the absolute quality of a single one, as well as the neural network. On the other hand, labeling a large number of samples with the help of some priori knowledge is easy if quality comparison can be modeled as a binary classification problem. In this case, labels are generated dynamically.

Inspired by RankIQA [47], the loss function of the IQA network is formulated as follows:

$$L_{QA}(I^{SR},I^{HR})=max(0,f(I^{SR})-f(I^{HR})+m)$$ (2)

where *f* (*I*^*SR*^) and *f* (*I*^*HR*^) are predicted values of *I*^*SR*^ and *I*^*HR*^, respectively. A higher value indicates better image quality. *m* stands for the margin, which adjusts the degree of punishment for fuzzy points near the boundary.

Eq (2) shows that if the prediction results are inconsistent with the actual ranking, then *f* (*I*^*SR*^) *> f* (*I*^*HR*^) *− m*, and the punitive steps should be performed. On the contrary, if the predictions truly reflect the actual ranking, then *f* (*I*^*SR*^) *≤ f* (*I*^*HR*^) *− m*, and the parameters shall not be updated.

Then, the self-supervised training of the IQA network is realized, solving the problem of label insufficiency.

Evidently, *m* in Eq (2) is a hyper-parameter and generally needs to be set manually. It would be elegant if its value can be adaptively adjusted. For further explanation, we define the discrimination of a network. For a pair of positive and negative samples, the following cases are considered: the outputs of network A are 0.9 and 0.1 and those of network B are 0.6 and 0.4. Then, we deem that A has higher discrimination ability than B. Combining the feature effectiveness and stability, it imposes stricter conditions on zero loss when *m* increases. The network is, then, forced to study the slight difference among samples, and the network is likely to possess relatively high discrimination when fully converged. The learning task can be difficult in this case, resulting in relatively slow convergence and less feature stability, which indicates that the IQA networks in adjacent phases tend to focus on different characteristics, causing an unsatisfactory jitter of the gradient descent direction. When *m* is small, the loss easily approaches zero. At this point, the goal is relatively simple and the network converges rapidly. The parameters of the IQA networks in the adjacent phases have a subtle difference from each other, and the given gradient descent direction remains consistent. Although the feature stability is enhanced, the effectiveness and the reference value of the feature decrease.

To obtain a tradeoff between the feature stability and feature effectiveness, we propose a dynamic adjustment strategy. The parameter *m* is dynamically adjusted during training, driving IQA to emphasize on the effectiveness in the early stage while on stability during the subsequent period. Therefore, the FR-IQA indicators that are negatively correlated to image quality are used to assess the margin to adjust the training targets dynamically. The IQA of the existing FR-IQA indicators is unreliable, and the contributions of the target adjustment on network training depend on the accuracy of the FR-IQA indicators to some extent. To weaken the effect caused by inconformity between FR-IQA indicators and human perception and to maintain a steady training, we take the moving average of the FR-IQA score as the margin.

To set the initial value of the margin, let

$$m_{0}=FRIQA(I_{0}^{SR},I_{0}^{HR})$$ (3)

For the *i*-th (*i >* 0) iteration, *m* is updated using

$$m_{i}=\beta \cdot m_{i-1}+(1-\beta )\cdot FRIQA(I_{i}^{SR},I_{i}^{HR})$$ (4)

where *m* is updated at each iteration (IQA and SR networks) to make a more precise approximation. Thus, the IQA loss function at the *i*-th iteration can be determined by the following:

$$L_{QA}{\left(I^{SR},I^{HR}\right)}_{i}=max(0,f(I^{SR})-f(I^{HR})+m_{i})$$ (5)

To better understand Eq (5), two extreme cases are analyzed. If *m* = *1*, then the loss function is summarized as follows:

$$L_{QA}{\left(I^{SR},I^{HR}\right)}_{m=1}=max(0,f(I^{SR})-f(I^{HR})+1)=(f(I^{SR})-0)+(1-f(I^{HR}))$$ (6)

Eq (5) degrades into the loss function for fitting problem, which classifies SR images to 0 and HR images to 1.

If *m* = *0*, then the loss function can be rewritten as follows:

$$L_{QA}{\left(I^{SR},I^{HR}\right)}_{m=0}=max(0,f(I^{SR})-f(I^{HR}))$$ (7)

Then, it can be viewed as a loss function for a binary classification problem.

In our work, the root mean square error (RMSE) and the perceptual index (PI) are used to evaluate the image distortion and perceived quality, respectively. The PI is calculated as follows:

$$PI=\frac{1}{2}((10-Ma)+NIQE)$$ (8)

where *Ma* and *NIQE* follow the same definition as in [8] and [52], respectively. For fair comparison, all reported RMSE and PI measures were calculated with the removal of four pixels from each border.

## 4. Experiments and analysis

To evaluate the performance of the proposed method, the networks were trained on the training set of DIV2K [53]. Then, comprehensive assessments of the proposed SISR model were carried out on several widely used benchmark databases, including DIV2K (we only used the first 16 images of the validation set due to high memory cost), PIRM-self [54], Set5 [55], Set14 [56], BSD100 [57], and Urban100 [58]. The IQA networks were pre-trained on the TID2013 dataset [59] and KonIQ10k dataset [60].

In this section, some basic settings of benchmarks for the experiment are provided, and then the details of the parameter selection are further described. Lastly, extensive comparison experiments, and quantitative analysis are also provided. We further compare our network to several state-of-the-art SISR methods. Our training was implemented in Pytorch 1.0.0 (Python 3.6) under Ubantu 16.04 operating system, and some tests were conducted in the MATLAB R2016a on an Intel i7-6700K (4.0 GHZ), GeForce GTX1080 with 16 GB RAM environment.

### 4.1 Network setup

#### SR Network setting

The parameters for the SR network were set as follows: the batch size is set to 16, and the training images are cropped into 48 *×* 48 non-overlapping patches to form the training samples. The weight coefficient is set as *w* = *{*0.3, 1*e*5, 1*e*5, 1*e*5, 0, 0*}*, and the total number of iterations is 1*e*5. The ADAM optimizer is used with the learning rate at 1*e −* 4, for both nets. For the IQA net, all the historical information of the gradient are cleared at the beginning of each phase. We fix the scaling factor at 4, and the FR-IQA metric in [38] is used to estimate the margin (*β* = 0.99).

#### IQA Network pre-training

We initially combined KonIQ10k dataset with TID2013 dataset to provide sufficient training samples. We trained our model with ADAM optimizer with the learning rate initialized as 1e − 4. We set the epoch size as 100. Simultaneously, we maintained the parameters of the third down-sampling layer and those ahead fixed, and the learning rate was reduced to 1e − 5 for fine tuning the parameters of the IQA network on Ma dataset [8]. Pre-training is necessary because it tunes the IQA network at an appropriate initial point, which effectively accelerates convergence.

### 4.2 Impact of SISR network parameters

#### Determination of *k* and *n*

To study the contributions of parameter *k* and *n* on the training effects, the number of iterations for a SR network is fixed at 60, 000, thereby ensuring that all SR networks are trained to the same extent. Let *r* = *k*/(*k* + *n*). When *k* is sufficiently large, the IQA network is sufficiently trained. Therefore, a larger *r* indicates that we focus more on feature effectiveness given that a more frequently updated network generally provides more up-to-date information, and a smaller *r* signifies that more focus is given on feature stability.

Although in exhaustive, the five listed data arrays show that: 1) the synchronous increase of *k* and *n* improves the assessment quality with fixed *r*. This finding is mainly caused by the SR net, which was trained more sufficiently, thereby enhancing the effectiveness and reliability of the extracted features. However, this result does not conclude that a larger *k* implies better performance. We have to reemphasize the influence of *r*. The comparative result among the 1*st*, 3*rd* and 5*th* sets of parameters provides some proof; 2) The results from the 1*st*, 3*rd* and 5*th* sets of parameters indicate that a noticeable change on the indices with different *r* values is found with fixed (*k* + *n*) and all *k* values at the same order of magnitude. This finding could possibly be explained by the different importance attached to the feature effectiveness and the feature stability. The 3*rd* set of parameters clearly shows the very small value of *r* results in insufficient effectiveness of feature representations, and the 5*th* set of parameters demonstrates that the large value of *r* can lead to poor stability of extracted features. Explicitly, the value of *r* has considerable performance implications.

Comparative experiments are conducted on 0812.*png* in DIV2K dataset to provide corresponding visual effect to elaborate the impact of the status of the IQA network on the training of the SR network intuitively.

Quantitative results on single-image DIV2K validation set are exhibited in Fig 4, where the pictures are restored using hyper-parameters from the first three groups in Table 1. The gradient instabilities cause reconstruction image artifacts using the first array of parameters. The reconstruction also suffers from excessive smoothing and color noise when the third group of parameters is selected. This finding is mainly induced by less effective feature representations. Although the result from the 2*nd* set of parameters executes a better PI performance than the first two sets, much longer time and more iterations (120, 000) are consumed for training than the 3rd set of experiments (100, 000 iterations). The experimental results also reflect that better recognition effect can be obtained through finer hyper-parameter tuning. As a compromise, *k* = 200 and *n* = 300 are set to achieve a better balance in terms of speed and accuracy.

**Fig 4:** The impact of IQA network’s status on the training of the SR network in vision. (a) is the result of 0812.*png* in DIV2K dataset using the 1*st* set of hyper-parameters, (b) is the result of 0812.*png* in DIV2K dataset using the 2*nd* set of hyper-parameters, (c) is the result of 0812.*png* in DIV2K dataset using the 3*rd* set of hyper-parameters.

**Table 1:** Effect of hyper-parameter on performance indicators.

NO.	Hyper-Parameters			Performance Indicators	
	*K*	*n*	*r*	*RMSE*	*PI*
1	1	1	0.5	10.7128	4.1245
2	500	500	0.5	11.3616	3.7267
3	100	400	0.25	10.2517	5.0542
4	200	300	0.4	10.7647	3.9531
5	300	200	0.6	10.8157	4.1707

#### Weight coefficients of losses

A total of 30 groups of parameters are tested to determine the weight coefficients of the different components of the loss function. In accordance with the weight of the perceptual loss, these parameters are again divided into three new groups, each of which contains 10 sets of different parameters. The weight coefficients of the three newly established groups are {1e^5^, 1e^5^, 1e^5^, 0, 0}, {2e^5^, 2e^5^, 2e^5^, 0, 0}, {4e^5^, 4e^5^, 4e^5^, 0, 0}. The weight coefficient of content loss for each group increases from 0.2 to 2 at a rate of 0.2.

The testing experiments are designed on PIRM-self [54] validation set that provides smaller image size and faster computing speed because calculating the evaluation index on DIV2K validation set is time consuming, and the result is shown in Fig 5. Nevertheless, model training is still conducted on the DIV2K validation set, which considers the identification of 30 datasets. The training iterations for different weight coefficient sets are considered 2*e*5 to reconcile with the training extent. Therefore, some results could have been over-fitted.

**Fig 5:** Comparisons of the performance curve of PI versus the RMSE in different weight coefficients of loss components.

The performance curve of PI versus the RMSE is shown in Fig 5. With RMSE in [11,12] and PI in [4.5, 5.5], the weight coefficients of the loss components slightly influenced the SR performance. This result also shows that our method is insensitive to the weight coefficients, thereby rendering great convenience in adjusting the SISR parameters.

### 4.3 Determination of margin m

We observed experimentally that the value of *m* fluctuates from 0.3 to 0.5 as the margin is estimated using MDSI [38]. To further highlight the enhancements of SR performance by margin estimation via FR-IQA metric, *m* takes on the value 0.3, 0.4, and 0.5. Meanwhile, the comparison experiment for various margins was conducted, and the results are listed in Table 2.

**Table 2:** Effect on method performance of different margin.

*m*	0.3	0.4	0.5	ma(MDSI)	ma(1-MSSSIM)
RMSE	10.5920	10.4720	10.4818	10.7647	**10.3405**
PI	4.1789	4.2518	4.3131	**3.9531**	4.4319

From the summary in Table 2, we can draw a clear conclusion that margin estimation through the moving average of MDSI effectively ameliorates network performance, thereby verifying the discussion in Section 3.3. In addition, comparisons between the last two columns in the table show that PI decreases using MS-SSIM, which demonstrates the significance of the FR-IQA metric selection to the result.

### 4.4 Comparison with other SR methods

Classical and the state-of-the-art SR methods, including Bicubic interpolation [61], EDSR [15], RCAN [17], EDSR-GAN [19], EDSR-VGG2,2 [24] and EnhanceNet [23], are compared with our model to demonstrate the superiority of the proposed method. To ensure fairness, the results of EDSR, RCAN, and EnhanceNet are obtained from the released codes. It should be pointed out that the architecture of SRGAN [19] is slightly adjusted when its model is replicated. To be specific, EDSR (It has been proved to have much better performance than the original SRResNet) is employed as the generator of SRGAN to exclude the influence of generators. To distinguish the original version from ours, the SRGAN in this work is marked as EDSR-GAN. EDSR net is also trained using MSE and VGG2,2 as the loss function respectively and represented as EDSR-VGG2,2. In addition, our method has been implemented separately by using EDSR and RCAN as the generator (SR net) and represented as Ours (EDSR) and Ours (RCAN), respectively.

#### 4.4.1 Quantitative comparison

On these basis, the, the above methods are quantitatively evaluated on the basis of RMSE and PI indicators, with datasets including PIRM-self, Set5, Set14, DIV2K, BSD100, and Urban100. Table 3 reports the corresponding results.

**Table 3:** Performance indicators of different methods on SR dataset with scale factor *×*4.

Method	PIRM-self	Set5	Set14	DIV2K	BSD100	Urban100
	(RMSE/PI)	(RMSE/PI)	(RMSE/PI)	(RMSE/PI)	(RMSE/PI)	(RMSE/PI)
Bicubic	16.9700/7.0010	17.3185/7.4664	18.5871/7.1970	13.3126/7.3138	17.7917/7.1880	24.8628/7.1584
EDSR	**11.1643**/5.2425	**6.8489**/5.7707	**11.1938**/5.3530	**8.8092**/5.6062	**12.5619**/5.3705	**15.3666**/5.1618
RCAN	**10.8312**/4.8312	**6.3941**/5.9163	**10.9239**/5.2332	**8.6054**/5.3651	**12.3545**/5.1393	**14.2759**/4.9794
EDSR-GAN	12.6563/3.216	8.5848/4.6989	12.7263/3.9112	10.0543/4.1310	13.7665/3.5843	17.3064/4.2103
EDSR-VGG2,2	11.8390/5.0593	7.4269 /6.3507	11.7883/5.3972	9.3512/5.2815	13.1319/5.7360	16.3068/5.0028
EnhanceNet	15.9853/**2.6876**	9.9432/**3.1410**	14.8162/**3.0091**	12.0428/**3.6170**	16.1286/**2.9794**	19.4939/**3.4054**
Ours(EDSR)	13.9166/3.0117	8.8144/**4.2492**	13.6566/3.6892	10.7607/**3.9532**	15.0210/3.1601	18.9136/3.6906
Ours(RCAN)	13.3740/**2.9748**	8.6329/4.7577	13.2347/**3.6012**	10.4531/4.1264	14.6446/**3.1214**	18.4560/**3.6458**

For convenience, the best two RMSE/PI values of each dataset are marked in bold and the next best RMSE/PI values are underlined. Table 3 clearly shows that RCAN achieves much lower RMSE than Bicubic and EDSR on all given test datasets. In particular, RCAN and EDSR have superior performance to Bicubic in RMSE and PI, thereby indicating less distortion and high perceptual quality. In addition, by comparing the results of RCAN and EDSR, the distortion can be further minimized when a deeper and more complex generator is assembled. However, none of the three methods provides a plausible and satisfactory PI, that is, the reconstruction results have poor or medium perceptual quality.

Considering the SR methods that emphasize perceptual quality, the approaches represented by EDSR-GAN, EDSR-VGG2,2, EnhanceNet, Ours(EDSR), and Ours(RCAN) have better performance in PI than the conventional method (*e*.*g*., Bicubic) and the MAE loss-based methods (*e*.*g*., RCAN and EDSR). Moreover, the ranking of RMSE is contrary to that of PI for perceptual loss-based SR methods that use generators with the same structures.

The results suggest that EDSR-VGG2,2 reaches the minimum RMSE together with the maximum PI, whereas an opposite effect could be observed for EnhanceNet. Our method gains satisfying RMSE and PI for both EDSR and RCAN generators. Therefore, the results suggest that our model achieves a good balance of AL and perceived quality. In addition, a horizontal comparison between Ours(EDSR) and Ours(RCAN) has been conducted on PIRM-self dataset. The comparison also shows that the improvement of generator structure will ameliorate the model performance, thereby coinciding with the conclusion in [62]. This finding also indicates the remarkable potential of our method for performance improvement.

Table 3 shows that the PI of Ours(EDSR) is superior to that of Ours(RCAN) on Set5 and DIV2K datasets. However, the result is very likely to be influenced by the specific distribution of data because the two datasets only contain 5 and 16 images, respectively. To exhibit the performance of our approach more intuitively, the scatter graph of RMSE versus PI, which presents the experimental results on PIRM-self in Table 3, is drawn in Fig 6.

**Fig 6:** Scatter graph of RMSE versus PI for our methods and others (Bicubic, EnhanceNet, EDSR, RCAN, EDSR-GAN, EDSR-VGG2,2), where a low PI value indicates better perceived quality and a small RMSE value indicates better absolute quality.

In Fig 6, the horizontal axis refers to PI, where a low PI value indicates better perceived quality; the vertical axis represents the RMSE, and a small RMSE value indicates better absolute quality. Contrary to RCAN, EnhanceNet displays excellent PI but poor performance in RMSE. Bicubic is disadvantaged in PI and RMSE because of the simple interpolation on LR images. However, these indicators of our methods are well situated on the plane, thereby further confirming that our model provides a compromise between perceptual quality and distortion measure.

#### 4.4.2 Visual effects comparison

The quantitative evaluation results of our models are provided on public benchmark datasets. Our models are compared with the state-of-the-art methods, including Bicubic, EDSR, RCAN, EDSR-GAN, EDSR-VGG2,2, EnhanceNet. For comparison, RMSE and PI for images on DIV2K, BSD100, Set5, Set14, and Urban100 datasets are measured with scale factor *×*4. Comparative results of visual effects are provided in Fig 7. The testing datasets used in Fig 7 were obtained from Huang [58] (https://github.com/jbhuang0604/SelfExSR).

**Fig 7:** Visual effects and quantitative comparison (RMSE and Perceptual Index) of our methods with Bicubic, EnhanceNet, RCAN, EDSR-GAN and EDSR-VGG 2,2. (a) shows the results of 095.png from Urban100 dataset, (b) shows the results of 039.png from BSD100 dataset, (c) shows the results of 001.png from Set5 dataset, (d) shows the results of 011.png from Set14 dataset, (e) shows the results of 804.png from DIV2K dataset, (f) shows the results of 805.png from DIV2K dataset, (g) shows the results of 057.png from Urban100 dataset, (h) shows the results of 080.png from Urban100 dataset, (i) shows the results of 801.png from DIV2K dataset.

Fig 7 visualizes the edge detail of the SR images. The networks trained with MAE Loss experience excessive smoothing and lack of physical realism. RCAN achieves slightly better performance than EDSR because of using an advanced network structure. Evidently, EDSR-VGG2,2 attains better visual experience than EDSR and RCAN. However, magnified images suffer from artifact that displeases visual experience. This finding is mainly caused by the max pooling layers of the VGG net. In addition, EnhanceNet obtains a satisfactory visual effect that embodies high-frequency distinct edge and abundant detail information. However, contrary to the feature distribution of natural images, high-frequency noise was unavoidably generated in the magnified images. This finding is particularly outstanding in Fig 7(b), which shows diminished visual impact in some cases.

In summary, EDSR-GAN achieves relatively better visual effect among various algorithms because its textual result approaches closer to the actual circumstance. Even so, EDSR-GAN is also over-smoothing and unable to restore the high-frequency details in some situations (Fig 7(d), 7(g) and 7(h)). Compared with EnhanceNet and EDSR-GAN, our method provides compromising yet competitive results. Our method is significantly better than EnhanceNet in terms of artifact and noise. Meanwhile, our method outperforms EDSR-GAN in terms of detailed information in some situations. In general, extensive benchmark experiments reveal that the proposed model achieves a better tradeoff between perceptual quality and distortion measure given that the performance is comparable to state-of-the-art methods.

#### 4.4.3. Complexity of networks parameters

In order to compare the network’s complexity of different algorithms, the number of network parameters is figured out and reported in Fig 8. Results are evaluated on Set5 with scale factor *×*4. In Fig 8(a), the horizontal axis refers to parameter number and the vertical axis represents the RMSE, while the horizontal axis shows parameter number and the vertical axis reflects PI in Fig 8(b).

**Fig 8:** Scatter graph of the number of parameters versus SR performance for our methods and others (Bicubic, EnhanceNet, EDSR, RCAN, EDSR-GAN, EDSR-VGG2,2). Results are evaluated on Set5 with scale factor ×4: (a) is the number of parameters versus RMSE, (b) is the number of parameters versus PI.

Through comprehensive analysis of Fig 8, it can be seen that the number of parameters of our network is identical to that of EDSR or RCAN since our method is on the basis of them. It has also demonstrated that the architecture proposed is opening, and thus not confined to a specific net model. The baseline of SR net is expected to be adjusted flexibly according to practical requirements. Under the same baseline, Ours(EDSR) achieves lower PI than that of EDSR-GAN with comparable RMSE. Although our method has no advantage in RMSE compared with EDSR-VGG2,2, the PI superiority is definite. The same conclusion can also be drawn on the comparison between Ours(RCAN) and RCAN. Overall, these results coincide with the conclusion of the previous quantitative and visual effects comparison.

## 5. Conclusion

In this paper, we propose an IQA-guided SISR method using DL networks. Taking into account of both absolute pixel loss and visual effects of the SR results, an improved IQA network is introduced to guide the adjustment of SR network parameters. To solve the problem of heterogeneous datasets used by IQA and SR networks, we establish an interactive training mechanism via cascaded network, where the IQA network acts as a supervisor when constructing loss function of the SR network. We also propose a pairwise ranking hinge loss method to overcome the shortcomings of insufficient samples during training process and prevent the over-fitting problems at the same time.

The performance comparison between our proposed method with recent SISR methods shows that the former achieves a better tradeoff between perceptual quality and distortion measure than the latter. To be specific, our proposed method has better performance in terms of artifact and noise. Meanwhile, our method outperforms others in terms of detailed information in some situations. Extensive benchmark experiments and analyses also prove that our method provides a promising and opening architecture for SISR, which is not confined to a specific network model.

Although the proposed method has achieved some good results, this work is just the beginning to implement this IQA-guided approach in SISR problem. In our work, the performance is proved through benchmark datasets, its robustness of different kinds of real data remains to be verified. In further works, we will develop this algorithm and make it applicable to more data types (such as infrared images, remote sensing images, et al.).

## Supporting information

S1 File (RAR)

S2 File (RAR)

S3 File (ZIP)

S4 File (ZIP)
